# Automated Breast Image Classification Using Features from Its Discrete Cosine Transform

**DOI:** 10.1371/journal.pone.0091015

**Published:** 2014-03-14

**Authors:** Edward J. Kendall, Matthew T. Flynn

**Affiliations:** Discipline of Radiology, Memorial University of Newfoundland, St. John's, Newfoundland and Labrador, Canada; University of Maryland, United States of America

## Abstract

**Purpose:**

This work aimed to improve breast screening program accuracy using automated classification. The goal was to determine if whole image features represented in the discrete cosine transform would provide a basis for classification. Priority was placed on avoiding false negative findings.

**Methods:**

Online datasets were used for this work. No informed consent was required. Programs were developed in Mathematica and, where necessary to improve computational performance ported to C++. The use of a discrete cosine transform to separate normal from cancerous breast tissue was tested. Features (moments of the mean) were calculated in square sections of the transform centered on the origin. K-nearest neighbor and naive Bayesian classifiers were tested.

**Results:**

Forty-one features were generated and tested singly, and in combination of two or three. Using a k-nearest neighbor classifier, sensitivities as high as 98% with a specificity of 66% were achieved. With a naive Bayesian classifier, sensitivities as high as 100% were achieved with a specificity of 64%.

**Conclusion:**

Whole image classification based on discrete cosine transform (DCT) features was effectively implemented with a high level of sensitivity and specificity achieved. The high sensitivity attained using the DCT generated feature set implied that these classifiers could be used in series with other methods to increase specificity. Using a classifier with near 100% sensitivity, such as the one developed in this project, before applying a second classifier could only boost the accuracy of that classifier.

## Introduction

Quality control systems have greatly improved the consistency of mammograms and technical advances have shortened exam time without negatively impacting performance [1]. The USA screening programs apparently operate at a sensitivity of 84.1% and a specificity of 90.4% [2]. Radiologist performance is an important component of program performance and no matter how skilled, reporting physicians will miss some cancers that, in retrospect, were visible in the mammogram [3]. Physician performance varies widely. One study reported a mean sensitivity of 77% with a range of 29% to 97%. In that study, specificity ranged from 71% to 99% with an average of 90% [3]. As may be expected, higher specificity and positive predictive value has been shown to correlate with more experience [3]–[5]. Double readings have been shown to significantly increase accuracy [6]–[9]. Sickles and colleagues [10] reported performance benchmarks based on an analysis of six breast cancer screening registries and more than 600 radiologists. Of particular interest, the abnormal findings rate was 8% and this was associated with a positive predictive value of 31.4%.

Various factors contribute to physician performance. Experience, specialized training and reading volume correlate with better performance [4]. Presentation difficulty is correlated with poorer performance, but readers disagree on what is a difficult presentation [11]. The reasons for screening misses are varied, but in one study the single largest factor was that patent evidence was overlooked [12]. This may be due to reader fatigue [13]. In addition, there is evidence to suggest that low prevalence predisposes screening radiologists to false negatives [14]. Prevalence appeared not to influence aggregate performance measures [15] but did negatively correlate with inter-observer variability [16] in that readers were more consistent in the clinical than in the laboratory environment. Evans and colleagues further investigated the prevalence effect [14].They were interested to learn if prevalence in breast screening resulted in a criterion shift as noted in other situations [17]. They found that false negative rates fell significantly as prevalence increased (12% high versus 30% low). On the other hand, the false positive rate did not differ significantly between the two states. Thus, it appears that increasing the prevalence of disease in the body of reviewed work may improve performance in the key false negative statistic.

A useful approach to improving detection is by enlisting a second reader. This is implemented in many reading centers. Alternatively, computer algorithms have been enlisted as second readers [8], [9], [18], [19]. The typical computer aided detection (CAD) approach includes a machine learning or training phase followed by pattern recognition and classification phase. When abnormalities are detected, they are marked for the radiologist's review. An inefficiency with this method is that many uninteresting objects may be marked, potentially reducing the specificity and increasing the time required for review [5], [20]–[22]. As a consequence, an increase in sensitivity may be accompanied by a decrease in specificity [5], [23].

An alternate approach to improving the efficiency of screening programs by pre-selecting higher likelihood cases has been reported [24]–[26]. Mammograms were transformed and filtered using a variety of wavelets. Features extracted from the resulting maps were used to remove low risk cases from further consideration. In one report this method provided near perfect sensitivity with greater than 60% specificity [26]. We postulated that discriminate use of the discrete cosine transform might provide useful classification features to identify normal mammograms.

This work was undertaken to improve breast screening program accuracy using automated classification. The goal was to determine if whole image features represented in the transform would provide a basis for binary classification, normal or suspicious. The overall approach taken consisted of four sequential steps. 1. Preprocessing, in which images were prepared by removing useless information and standardizing size, resolution, and bit depth. 2. Transformation- Images were cosine transformed to arrange image data by spatial frequency in two dimensions. 3. Feature extraction- A small group of values were calculated from the transform for each image. 4. Classification- Machine learning was used to classify images by comparing them with images of known pathology. The output would be two pools, one containing normal and the other suspicious images. If successful the pool containing suspicious images would be enriched in cancer positive cases and subsequent interpretation achieve a lower false negative rate.

## Materials and Methods

Programs for this work were developed in Mathematica version 8.0. Input data was obtained from two publicly available mammographic image databases. The Digital Database for Screening Mammography (DDSM) [27], [28] and the Mammographic Image Analysis Society (MIAS) databases [29]. Both included “ground truth” data that describes the type and location of abnormalities present in the images. Images were extracted, rescaled to 200 μm resolution and padded or cropped to 1024^2^ pixels.

The subset of the MIAS database used in this study consisted of 205 normal, 54 benign cases and 41 malignant cases all in the mediolateral oblique (MLO) view. The DDSM medial lateral oblique (MLO) view data subset consisted of 269 normal, 70 suspicious (5 benign cases and 65 malignant) cases and the DDSM cranio-caudal (CC) view data subset contained 278 normal, 73 suspicious (5 benign cases and 68 malignant) cases.

Artifacts such as orientation tags were removed using a large-bright-object binary mask based on peak separation in the intensity histogram. Half-mean or mean value provided the best discrimination. The Hadamard product of the mask and the original image produced an image containing only the relevant breast tissue.

Frequency space maps were generated using the discrete cosine transform. In these, data were partitioned into L-shaped blocks, each twice the width of the proceeding block. The DC coefficient and the mean, standard deviation, skewness, and kurtosis determined for each of the ten blocks in the map, provided 41 features per map.

Two classification approaches were tested, k-nearest neighbor (KNN) and naive Bayesian.

### K-nearest neighbor

The twenty-five closest neighbors to each image feature were stored in the database as was their ordering and their fractional distance (d/d_max_). Combinations of two and three features were also tested.

Vote taking was used to determine classification. Votes were unweighted or weighted according to distance and/or prior probability. The algorithm was tested for between 1 and 25 calculated neighbors for each test image using the leave-one-out cross validation. The classification was found by adding the values assigned to the first k neighbors for each image. Suspicious images were assigned a vote value of +1 (x weighting) and normal images were assigned a vote value of −1 (x weighting). Adding the votes resulted in a value greater than or equal to zero if the consensus was suspicious and less than zero if normal.

Twelve variations of the classifier were calculated. For each variation, and each number of neighbors, the feature vector with the highest sensitivity was selected and recorded along with its specificity.

### Naive Bayesian classifier

For the naive Bayesian classifier, the program ran in two stages. First, posterior probabilities for all forty-one features were calculated. Next, these were compared with truth-data to determine the sensitivity and specificity of each feature.

Identically binned feature-histograms for normal and suspicious images were established. These were populated with the images according to their feature value. The number of normal and suspicious images in each bin provided the probability value for that feature value. Next each image feature was tested using leave-one-out cross validation.

The likelihood that the test image was suspicious (or normal) was calculated as likelihood_suspicious_  =  (suspicious counts)/(total suspicious).

Posterior probabilities (PP) were calculated as the likelihoods (suspicious or normal) multiplied by the corresponding prior probabilities. Suspicious posterior probability was normalized to the sum of the normal and suspicious posterior probability. The normalized posterior probability that an image was suspicious was then added to the database.

The whole process was repeated for all images in the set, for each feature and using between two and 20 bins. This process was repeated using combinations of two and three features (820 and 10660 possible combinations). For each additional feature added, separate histograms were generated and likelihoods calculated.

Once the database was populated with probabilities for each image for every possible combination of one, two, and three features, then sensitivity and specificity were calculated. In order to determine if an image was deemed suspicious, a certain suspicious-threshold probability had to be chosen, above which the image would be classified as suspicious. Since the classifications of images in the training set were known and all posterior probabilities were calculated, thresholds were chosen based on this data.

For 100% sensitivity, the lowest probability of a suspicious image being suspicious was used as the threshold. Specificity was then incrementally increased by using the second lowest probability of a suspicious image being suspicious as the threshold. Sensitivity and specificity were calculated for various threshold values in order to generate ROC data for each experimental setup. Optimal setup parameters were determined using the single feature classifier.

Statistical comparisons were performed for ROC curves following the methods of Delong [30]. Paired and unpaired t-tests were performed as appropriate.

## Results

Two classification engines were examined, k-nearest neighbor and Bayesian. In both cases, various conditions were investigated to determine each engine's optimal performance. This data is reported in the following sections.

### k-nearest neighbor

#### Determining the best features

Testing the MIAS, DDSM MLO and DDSM CC datasets using single feature classifiers for between 1 and 25 neighbors took on the order of minutes for each set. For each of the 12 variants of the classifier, the most sensitive feature or feature set was recorded with its corresponding specificity (not shown). For MIAS the three best features (sensitivity values in brackets) were block 2 skewness (16.8%), block 2 kurtosis (21.9%), and block 1 standard deviation (39.4%). For DDSM MLO the three best features were block 3 skewness (19.1%), block 4 mean (26.7%), and block 2 standard deviation (42.0%). For DDSM CC the three best features were block 6 kurtosis (10.8%), block 1 kurtosis (21.9%), and block 3 skewness (69.1%). In each trial using a combination of three features provided the best results.

#### Trial 1: Unweighted majority voting

The first variant of the k-nearest neighbor classifier assigned all votes an identical weight. For each data set, the best sensitivity was found using two neighbors and three features (Table 1). This configuration achieved 69.5% sensitivity and 51.7% specificity for MIAS, 82.9% sensitivity and 78.8% specificity for DDSM MLO and 83.6% sensitivity and 80.9% specificity for DDSM CC. The positive predictive value (PPV) ranged from 35 to 52% and the negative predictive value (NPV) from 78 to 95% (Table 1). This classifier trended toward higher specificity and lower sensitivity (Figure 1) as the number of neighbors included increased.

**Figure 1:** Unweighted KNN classifier. Sensitivity (Sen, solid lines) and specificity (Sp, dashed lines) versus Number of Neighbors for all three datasets. MIAS (red), DDSM MLO (green), DDSM CC (black).

**Table 1:** KNN classifier performance.

Data	No. of Neighbors	Distance weighting	Prior Probability Weighting	Sensitivity (%)	Specificity (%)	PPV	NPV
MIAS	2	N	N	69.5	51.7	0.40	0.78
DDSM (MLO)	2	N	N	82.9	78.8	0.35	0.92
DDSM (CC)	2	N	N	83.6	80.9	0.52	0.95
MIAS	1 or 2	Y	N	51.6	72.2	0.47	0.76
DDSM (MLO)	3	Y	N	65.7	85.1	0.53	0.91
DDSM (CC)	5	Y	N	61.6	89.6	0.61	0.90
MIAS	3	N	Y	83.2	34.6	0.37	0.81
DDSM (MLO)	13	N	Y	98.6	63.2	0.41	0.99
DDSM (CC)	23	N	Y	98.6	75.2	0.51	1.00
MIAS	2	Y	Y	69.5	52.5	0.41	0.79
DDSM (MLO)	15	Y	Y	98.6	65.7	0.43	0.99
DDSM (CC)	12	Y	Y	97.3	75.9	0.51	0.99

Note. The factors were tested using the best three features for each dataset.

#### Trial 2: Distance weighted votes

Using votes weighted by distance, the best sensitivities were found using three features (Table 1). For the MIAS set, the highest sensitivity was 51.6% with 72.2% specificity. For the DDSM MLO set, the best performance was 65.7% sensitivity and 85.1% specificity for 3 neighbors. For the DDSM CC set, the best performance obtained was 61.6% sensitivity and 89.6% specificity for 5 neighbors. This classifier achieved a PPV ranging from 47 to 51% and an NPV ranging from 76 to 91%. With more neighbors, the sensitivity and specificity diverge further, with the effect most pronounced in the MIAS set (Figure 2).

**Figure 2:** Distance weighted KNN classifier. Sensitivity (Sen, solid lines) and specificity (Sp, dashed lines) versus Number of Neighbors for all three datasets. MIAS (red), DDSM MLO (green), DDSM CC (black).

#### Trial 3: Prior probability weighted votes

With votes adjusted for the prior probabilities (Table 1). For MIAS the highest was 92.7% sensitivity and 39.0% specificity with 6 neighbors. For DDSM MLO the highest was 98.6% sensitivity and 63.2% specificity with 13 neighbors. For DDSM CC the highest was 98.6% sensitivity and 75.2% specificity with 23 neighbors. The classifier achieved a PPV range from 37 to 51% amd an NPV range from 81 to 100%. Unlike the first two classifiers, this one favored sensitivity over specificity (Figure 3).

**Figure 3:** Prior probability weighted KNN classifier. Sensitivity (Sen, solid lines) and specificity (Sp, dashed lines) versus Number of Neighbors for all three datasets. MIAS (red), DDSM MLO (green), DDSM CC (black).

#### Trial 4: Distance weighted and prior adjusted voting

When using both distance weighting and prior probabilities, the best classifiers used three features (Table 1). For MIAS the highest was 85.4% sensitivity and 55.1% specificity with 24 neighbors. For DDSM MLO, the highest was 98.6% sensitivity and 65.7% specificity with 15 neighbors. For DDSM CC, the highest was 97.3% sensitivity and 75.9% specificity with 12 neighbors. The classifier provided a PPV range of 41 to 51% and an NPV range of 79 to 99%. Weighting by neighbor distance, did not have a significant positive effect on the performance of the classifiers.

### Bayesian classification

The naive Bayesian classifier was tested for all data sets using 1, 2 and 3 features and 2 to 25 histogram bins. The classification histograms were optimized at 12 bins for MIAS and DDSM MLO and 13 bins for the DDSM CC data. Thresholds were adjusted to generate ROC curves.

### Best performing features at 100% sensitivity

For the MIAS data set, the best performing features were: block 3 kurtosis, for one feature classifiers, DC offset and block 3 kurtosis for two feature classifiers, and DC offset, block 1 skewness and block three kurtosis for three feature classifiers.

For the DDSM MLO data set, the best performing features were block 4 mean for one feature classifiers, block 4 mean and block 3 skewness for two feature classifiers, and block 2 standard deviation, block 2 skewness, and block 3 skewness for three feature classifiers.

Finally, for the DDSM CC data set, the best performing features were: block 2 standard deviation for one feature classifiers, block 2 standard deviation and block 3 skewness for two feature classifiers, and block 4 mean, block 2 standard deviation, and block 3 skewness for three feature classifiers.

### Feature vector size

Figure 4 shows the specificity achieved for each of the data sets using one, two, or three features. Two feature classifiers performed better than one, and generally three feature classifiers performed better than two. However, there were diminishing gains with the third added feature.

**Figure 4:** Effect of feature vector size on Bayesian classifier performance. Specificity versus sensitivity for all datasets. One (light grey), two (medium grey) or three (dark grey) feature combinations were tested at three sensitivity levels.

Using a Bayesian classification scheme permits adjusting its performance on the training set. When the sensitivity was adjusted (97–98%) to allow a few false negative images, specificity increased by 2 percentage points for MIAS, 9 percentage points for MLO and 15 percentage points for the CC data set (Table 2). The PPV for MIAS did not change but that of MLO increased by 7 percentage points and that of CC increased by 11 percentage points. The NPV declined by 4 percentage points for MIAS and 1 percentage point for MLO and CC data sets. After classification, the MIAS suspicious data sets had a 15% increased disease prevalence and disease doubled in the MLO and CC data sets.

**Table 2:** Bayesian classifier performance^a^.

Data	Sensitivity (%)	Specificity (%)	PPV	NPV	Prevalence Gain^b^
MIAS	1.00	0.19	0.37	1.00	1.15
MIAS	0.99	0.20	0.37	0.98	1.15
MIAS	0.98	0.21	0.37	0.96	1.16
DDSM (MLO)	1.00	0.64	0.42	1.00	2.04
DDSM (MLO)	0.99	0.72	0.48	0.99	2.32
DDSM (MLO)	0.97	0.73	0.49	0.99	2.35
DDSM (CC)	1.00	0.62	0.41	1.00	1.97
DDSM (CC)	0.99	0.76	0.52	1.00	2.51
DDSM (CC)	0.97	0.77	0.53	0.99	2.54

a Classification was performed using the best three features for each dataset.

b Prevalence gain  = TP/(TP+FP)_c_/TP/(TP+FP)_o_ is the fractional increase of truly positive images in the suspicious classification.

#### Overall accuracy

The best classified data sets were the DDSM MLO and DDSM CC. They performed far better than the smaller MIAS set.

Receiver operating characteristic (ROC) curves were calculated for all the datasets using one, two or three features. In all cases classification was better than random. Figure 5 provides the results when three features were used in the classification. The number of features used in classification did not significantly alter the ROC response within each dataset (Table 3). The MIAS set produced the poorest performance (Figure 5). The DDSM MLO and CC datasets offered better classification and did not differ significantly from each other (Table 3). The MIAS performance differed significantly from that of the other two datasets (Table 3).

**Figure 5:** Bayesian three feature classifier performance. Sensitivity versus 1-specificity. The performance of the classifier was tested on MIAS (red), DDSM CC (blue and DDSM MLO (black) datasets. as was the case for one and two features the algorithm performed much better on the CC and MLO datasets.

**Table 3:** Bayesian Classifier Performance.

	MIAS-1^a^	MIAS-2	MIAS-3	DDSM-MLO-1	DDSM-MLO-2	DDSM-MLO-3	DDSM-CC-1	DDSM-CC-2
MIAS-2	−1.10^b^							
MIAS-3	−1.07	0.04						
DDSM-MLO-1	−5.74	−4.60	−4.64					
DDSM-MLO-2	−6.92	−5.74	−5.78	−1.01				
DDSM-MLO-3	−7.46	−6.27	−10.03	−1.47	−0.47			
DDSM-CC-1	−6.06	−10.07	−4.95	−0.25	0.77	1.24		
DDSM-CC-2	−6.92	−5.74	−5.78	−0.99	0.02	0.50	−0.75	
DDSM-CC-3	−7.38	−6.18	−6.22	−1.38	−0.37	0.10	−1.14	−0.40

Comparison of ROC curves.

a 1,2 and 3 refer to the number of features used in the classification.

b the t-statistic was calculated using the method described by Delong and colleagues (20). Values less than1.96 indicate no significant difference in the comparison.

At 100% sensitivity, for DDSM MLO with a three feature classifier, 64.3% specificity was obtained. In other words 173 normal images may be removed from the set of 339 images.

## Discussion

The ability of features derived from a discrete cosine transform (DCT) of mammograms to distinguish normal from suspicious breast images was tested in three datasets.

The algorithms were adjusted to get the best possible accuracy for MIAS (sensitivity of 100% and a specificity of 19.0%). When the DDSM MLO set was introduced, using the exact same algorithm, there was a substantially better performance (sensitivity of 100% and a specificity of 64.3%). Since the DDSM subset used here was only slightly larger than the MIAS, size probably did not have a significant impact. However, the datasets were qualitatively different. In the MIAS set, 60 of the 95 suspicious images were benign, whereas in the DDSM set only 5 of the 70 suspicious images were benign. Furthermore, all five of those benign findings were contralateral to a malignant image. In a separate experiment a new data set will be created to determine if the benign findings rate degrades the separation of normal from suspicious images.

Choosing the best classifier is often an arbitrary exercise [5]. Here, since a false negative might have severe health repercussions, features and classifiers with the highest sensitivities were chosen as “best”. Choosing classifiers with the highest sensitivity provided a consistent basis of comparison.

In this study neither the KNN nor the naive Bayesian classifiers emerged as superior under all conditions. However, the naive Bayesian classifier had some favorable characteristics. For example, as an eager learner, it had a more efficient operational phase. Since all that needed to be taken from the training phase were two histograms per feature, storage requirements were low. In addition, computational requirements for classification were low. The k-nearest neighbor classifier on the other hand required the feature values and classifications for all images in the training set to be saved, requiring more storage. Classification of each new image required comparison to every image in the training set before votes could be tabulated.

The naive Bayesian classifier is also quite flexible. The threshold of what to consider normal and what to consider suspicious can be changed without having to retrain the classifier. This allows the selection of how much emphasis to place on sensitivity and how much to trade off for increased specificity. An adjustable KNN classifier could be developed by changing the weighting assigned to suspicious and normal neighbor votes. As seen for the prior adjusted results though, this produces some odd behavior in the classifier depending on the number of neighbors used (Figures 1–3).

The classifiers used no more than three features. Despite this small feature vector size, the results were still quite accurate. Using such a small number of features ensured that over training would not be an issue. The consistent high performance of these features for different data sets and different classification algorithms suggests that the high classification rates are due more to the features themselves than to the classifiers or to random chance.

The high sensitivity attained using the DCT generated feature set means that one of the classifiers developed in this project could be used in series with other computer aided detection methods to increase overall accuracy [31]. Using a classifier with near 100% sensitivity, such as the one developed in this project, before applying a second independent classifier may boost the overall accuracy. At 100% sensitivity, no suspicious images are lost, while some (64% in the case of naive Bayesian classification of DDSM MLO) of the normal images can be removed to a separate low priority processing queue. In the high priority queue, the second classifier is given a smaller group of images that are more likely to be suspicious.

It appears that the DCT feature based classifiers performance is in the useful range [10]. Sickles and colleagues have provided reference values to compare the performance of mammographic stations [10]. If we assume that their published PPV mean values have a normal distribution, the performance of the KNN and Bayesian classifiers here is significantly better than these benchmarks.

This classifiers had two outputs, one that contained only normal images and the other contained normal and suspicious images. The algorithm allows selection of a sensitivity threshold. Disease prevalence in output one can be zero or can be detuned to allow false negatives. In the first instance, all of the suspicious images are in output two. If this output was referred to a mammographer the performance obtained may approximate that described by Evans and colleagues [14]. They claim that interpretation performance improves when disease incidence increases. At the very least, triaging the exams into high an low priority streams may reduce reader fatigue, a factor thought to contribute to false negative findings[13]. Investigations are underway to determine the extent of enrichment possible in a contemporary clinical setting and if that enrichment results in a lower false negative rate.
